The article "Comparing Outcomes between Major Trauma Patients Transferred from a Different Hospital and Patients Transported Directly to Trauma Centers: A Retrospective Analysis with Propensity Score Matching Analysis" was published in 2022. Journal: Emerg Med Int.

# Comparing Outcomes between Major Trauma Patients Transferred from a Different Hospital and Patients Transported Directly to Trauma Centers: A Retrospective Analysis with Propensity Score Matching Analysis

**DOI:** 10.1155/2022/4430962

**Published:** 2022-08-02

**Authors:** Cheng-Hsi Yeh, Sheng-En Chou, Wei-Ti Su, Ching-Hua Tsai, Chun-Ying Huang, Shiun-Yuan Hsu, Ching-Hua Hsieh

**Affiliations:** ^1^Department of General Surgery, Kaohsiung Chang Gung Memorial Hospital and Chang Gung University College of Medicine, Kaohsiung 83301, Taiwan; ^2^Department of Trauma Surgery, Kaohsiung Chang Gung Memorial Hospital and Chang Gung University College of Medicine, Kaohsiung 83301, Taiwan

## Abstract

This study aimed to explore differences in outcomes between these major trauma patients who were transferred and those directly transported to trauma centers. The medical information and outcome of 5,341 major trauma patients with an injury severity score (ISS) ≥ 16 who were hospitalized for treatment between January 1, 2009, and December 31, 2019, were collected from the Trauma Registry System of the hospital. There were 2,386 patients who were transferred (transfer group) and 2,955 patients transported directly to trauma centers first (direct group). Regarding the outcomes, there was no significant difference in the mortality rate between patients in the transfer group and the direct group (11.1% vs. 10.5%, respectively, *p*=0.527). However, the patients in the transfer group had a longer hospital stay (16.8 days vs. 14.3 days, respectively, *p* < 0.001) and higher incidence of intensive care unit (ICU) admission (74.9% vs. 70.5%, respectively, *p* < 0.001) than those patients in the direct group. Similar results were observed in the selected 2,139 pairs of propensity score-matched patient populations, who did not present with significant differences in sex, age, comorbidities, trauma mechanisms, and ISS. This study revealed no significant difference in the mortality rate between the two groups of major trauma patients. However, the transferred patients had significantly longer hospital stays and higher rates of ICU admission than patients directly transported to trauma centers.

## 1. Introduction

It is estimated that about 5.8 million people die from trauma every year, accounting for 10% of the world's deaths [1]. To improve outcomes and decrease morbidity and mortality, timely and appropriate resuscitation of patients with major trauma is vital [2, 3]. Transporting patients with major traumas directly to trauma centers has been suggested to be more beneficial than transporting to non-trauma centers [4–6]. For example, a report from England revealed that, when compared with patients that were directly transferred to a trauma center, secondary transfer of the patients for definitive care was associated with significantly delayed imaging, delayed surgery, and increased mortality in major trauma patients [7]. A similar US study revealed increased craniotomy, hospital stay, and mortality among patients transferred to non-trauma centers [8]. However, some authors claimed that immediate resuscitation played a more important role, regardless of where the patients were taken for definitive care [9]. Therefore, we set out to study the issue regarding whether there was a different outcome between those major trauma patients who were transferred and those transported directly to trauma centers. In addition, it has been reported that unadjusted prehospital confounding factors influence the evaluation of the impact of transport directness on mortality outcomes [10]. Herein, under the use of propensity score matching to attenuate the baseline difference in demographic and injury characteristics of the study populations, the primary aim of this study is to assess the mortality outcomes between the major trauma patients who were transferred and those directly transported to trauma centers. The secondary aim is to compare the length of hospital stay and the rate of intensive care unit (ICU) admission of these patients in both groups.

## 2. Methods

### 2.1. Ethics Statement

This study was approved by the Institutional Review Board (IRB) of Chang Gung Memorial Hospital (approval number: 202002038B0). Because the study was designed for retrospective analysis of the registered database, the need for informed consent was waived according to IRB regulations.

### 2.2. Patient Population and Retrieved Information

After the selection from the enrolled 39,135 hospitalized trauma patients injured by all trauma causes for treatment between January 1, 2009, and December 31, 2019 (Figure 1), there were 2,386 patients who had major trauma, defined as an injury severity score (ISS) ≥ 16, in the transfer group and 2,955 major trauma patients in the direct group. The following patient information was collected from the Trauma Registry System of the hospital: sex, age, and preexisting comorbidities (cerebral vascular accident (CVA), hypertension (HTN), coronary artery disease (CAD), congestive heart failure (CHF), diabetes mellitus (DM), and end-stage renal disease (ESRD)); mechanism of trauma (automobile accident, motorcycle accident, bicycle accident, pedestrian, fall accident, penetrating injury, and strike by/against injury), Glasgow Coma Scale (GCS) score, systolic blood pressure (SBP), heart rate (HR), and respiratory rate (RR) upon arrival to the emergency room; cardiopulmonary resuscitation, need for intubation, chest tube insertion, and blood transfusion performed in the emergency room; abbreviated injury scale (AIS); ISS; in-hospital mortality; hospital stay (days); and admission to the ICU.

### 2.3. Statistical Analysis

The distribution data for continuous variables were normalized using the Kolmogorov–Smirnov test. Analysis of variance (ANOVA) was used with Bonferroni post hoc correction to analyze continuous data with normal distribution, and the results were expressed as mean ± standard deviation (SD). Non-normally distributed continuous data were analyzed using the Mann–Whitney *U test*. The results are expressed as mean ± SD or median with interquartile range (IQR, Q1–Q3). Categorical data were compared using two-sided Fisher's exact or Pearson *χ*^2^ test, with odds ratios (ORs) and 95% confidence intervals (CIs). To attenuate the baseline difference of the patients in both groups because of non-random assignment of the patients, we established a 1 : 1 propensity score-matched study group using the greedy method with a 0.2 caliper width to compare the outcomes of these patients in the transfer group with the patients in the direct group. The in-hospital mortality of patients was defined as the primary outcome. The length of hospital stays and the requirement for ICU admission were defined as secondary outcomes. All statistical analyses were performed using SPSS (version 23.0; IBM Inc., Chicago, IL, USA). Statistical significance was set at *p* < 0.05.

## 3. Results

### 3.1. Demographic and Injury Characteristics of the Patients with Major Trauma

The patients in the transfer group were predominantly younger men, had fewer comorbidities of CVA, HTN, DM, and ESRD, and sustained a higher incidence of automobile and motorcycle accidents but a lower incidence of fall accidents than those in the direct group (Table 1). Patients in the transfer group had a lower GCS level, higher incidence of AIS ≥2 in the regions of the thorax, abdomen, and extremities, and higher ISS than the patients in the direct group. There was no significant difference in the mortality rate between patients in the transfer group and the direct group (11.1% vs. 10.5%, respectively, *p*=0.527). However, the patients in the transfer group had a longer hospital stay (16.8 days vs. 14.3 days, respectively, *p* < 0.001) and higher incidence of ICU admission (74.9% vs. 70.5%, respectively, *p* < 0.001) than those in the direct group.

### 3.2. Physiology and Procedures Performed on the Major Trauma Patients at the ER

Regarding the presenting physiology at the ER (Table 2), patients in the transfer group had a higher incidence of GCS < 13 and HR > 100 beats/min, but a lower incidence of having RR < 10 or >29 breaths/min than those in the first group. There were no significant differences in the incidence of SBP < 90 mm·Hg between the two groups. Regarding the procedures performed at the ER, the patients in the transfer group had a significantly lower incidence of receiving cardiopulmonary resuscitation, intubation, and chest tube insertion than those in the direct group.

### 3.3. Comparison of Outcomes between the Propensity Score-Matched Patients in the Transfer and Direct Groups

A 1 : 1 propensity score-matched patient cohort was created for patients in the transfer group compared to those in the direct group to attenuate the confounding effects of the patients' baseline characteristics on outcome measurements (Table 3). The selected 2,139 pairs of propensity score-matched patient populations, who did not present with significant differences in sex, age, comorbidities, trauma mechanisms, and ISS, showed no significant difference in the in-hospital mortality rate between the transfer group and the direct group (*p*=0.314). However, the patients in the transfer group still had significantly longer hospital stay (16.6 days vs. 14.7 days, respectively, *p* < 0.001) and ICU admission rate (73.9% vs. 70.9%, respectively, *p*=0.026) than the direct group of patients.

## 4. Discussion

This study revealed that, in Taiwan, there was no significant difference in the mortality rate between patients with major trauma injuries who were transferred from other hospitals and those transported directly to trauma centers for definitive care; this result was found in both the study population and in the 1 : 1 propensity score-matched patient cohorts. This is contradictory to some US studies which demonstrated that patients with major trauma taken directly to a trauma center had lower mortality than those seen at other hospitals and subsequently referred to a trauma center for definitive care [4, 11]. In Taiwan, most traffic accidents are motorcycle accidents that occur in relatively crowded streets, and the transport times of patients to the emergency room are short (average 12 min for Taipei according to government data [12] and 18 min for Kaohsiung according to our previous analysis) [13, 14]. Therefore, we believe that the short transportation time from the accident scene to the emergency room may partly explain why there was no significant difference in the mortality rate between the patients who were transferred from other hospitals and those transported directly to trauma centers first. This result may also imply the importance of immediate resuscitation instead of the hospital the patient is sent [9].

However, the patients in the transfer group had a significantly longer hospital stay and ICU admission rate than the patients in the direct group. This result is in accordance with reports by Young et al. that demonstrated that patients with major trauma taken directly to a trauma center had shorter hospital stays than those seen at other hospitals and subsequently referred to the trauma center [11]. The reason for the longer hospital stay and a higher rate of ICU admission may be reasonable, as some studies reported that transfer for the patients might delay the definite management for surgical intervention such as spinal cord injury [15], emergency general surgery [16], or hip fracture surgery [17] and some physicians may prefer an ICU admission, with a subsequent longer stay, for transferred patients [18]. However, the indications for ICU admission or discharge of the patients were unknown and may vary among different physicians; therefore, some selection bias may exist in the interpretation of the data.

This study had some limitations. First, there may have been selection bias in the retrospective design of this study. Second, the patients declared dead on arrival at the emergency room and the potential transfers were not recorded in the registered database, and only in-hospital mortality, but not long-term mortality, was evaluated in this study. Both conditions may have led to a selection bias in the mortality outcome measurement. Third, the indication for transfer is unknown, and another selection bias may exist because the patients recovered at the regional hospital without transfer. Furthermore, interventions such as resuscitation, damage control, and surgery could lead to a different outcome for the patients; however, in this study, we can only assume that the outcome of these interventions was uniform across the studied population in various hospitals. Finally, the population included in this study was limited to a single urban trauma center; thus, these results may not be generalizable to other regions.

## 5. Conclusions

This study revealed no significant difference in the mortality rate between the major trauma patients who were transferred from other hospitals and those transported directly to trauma centers. However, the patients that underwent transfer to a trauma center for definitive care had significantly longer hospital stays and higher rates of ICU admission than patients transported directly to trauma centers.

## Figures and Tables

**Figure 1:** Flowchart illustrating the inclusion of adult patients with major trauma from the Trauma Registry System, with the allocation of these patients into transfer (transferred patients) and direct groups (visited the hospital firstly).

**Table 1:** Demographic and injury characteristics of the trauma patients with injury severity score equal to or more than 16.

Variables	Transfer (*n* = 2,386)	Direct (*n* = 2,955)	OR (95% CI)	*p*
Gender				<0.001
Male, *n* (%)	1630 (68.3)	1848 (62.5)	1.3 (1.15–1.45)	
Female, *n* (%)	756 (31.7)	1107 (37.5)	0.8 (0.69–0.87)	

Age (years)	54.2 ± 19.3	57.8 ± 18.9	—	<0.001

Comorbidities				
CVA, *n* (%)	82 (3.4)	189 (6.4)	0.5 (0.40–0.68)	<0.001
HTN, *n* (%)	738 (30.9)	1019 (34.5)	0.9 (0.76–0.96)	0.006
CAD, *n* (%)	128 (5.4)	177 (6.0)	0.9 (0.70–1.12)	0.328
CHF, *n* (%)	12 (0.5)	14 (0.5)	1.1 (0.49–2.30)	0.879
DM, *n* (%)	389 (16.3)	553 (18.7)	0.8 (0.73–0.98)	0.022
ESRD, *n* (%)	51 (2.1)	92 (3.1)	0. 7 (0.48–0.96)	0.028

Trauma mechanisms				
Automobile, *n* (%)	149 (6.2)	58 (2.0)	3.3 (2.44–4.53)	<0.001
Motorcycle, *n* (%)	1340 (56.2)	1463 (49.5)	1.3 (1.17–1.46)	<0.001
Bicycle, *n* (%)	111 (4.7)	126 (4.3)	1.1 (0.84–1.42)	0.493
Pedestrian, *n* (%)	82 (3.4)	128 (4.3)	0.8 (0.59–1.04)	0.094
Fall, *n* (%)	608 (25.5)	1065 (36.0)	0.6 (0.54–0.68)	<0.001
Penetrating injury, *n* (%)	7 (0.3)	12 (0.4)	0.7 (0.28–1.84)	0.492
Strike by/against, *n* (%)	89 (3.7)	103 (3.5)	1.1 (0.80–1.43)	0.633
GCS, median (IQR)	15 (8–15)	15 (11–15)	—	<0.001
3–8, *n* (%)	611 (25.6)	505 (17.1)	1.7 (1.46–1.91)	<0.001
9–12, *n* (%)	261 (10.9)	330 (11.2)	1.0 (0.82–1.16)	0.791
13–15, *n* (%)	1514 (63.5)	2120 (71.7)	0.7 (0.61–0.77)	<0.001

Injury regions with AIS ≥2				
Head/neck, *n* (%)	1888 (79.1)	2398 (81.2)	0.9 (0.77–1.01)	0.065
Face, *n* (%)	432 (18.1)	512 (17.3)	1.1 (0.92–1.22)	0.458
Thorax, *n* (%)	761 (31.9)	862 (29.2)	1.1 (1.01–1.28)	0.031
Abdomen, *n* (%)	383 (16.1)	371 (12.6)	1.3 (1.14–1.55)	<0.001
Extremity, *n* (%)	904 (37.9)	998 (33.8)	1.2 (1.07–1.34)	0.002
ISS, median (IQR)	20 (16–25)	20 (16–25)	—	<0.001
16–24, *n* (%)	1644 (68.9)	2177 (73.7)	0.8 (0.70–0.89)	<0.001
≥25, *n* (%)	742 (31.1)	778 (26.3)	1.3 (1.12–1.42)	<0.001
Mortality, *n* (%)	264 (11.1)	311 (10.5)	1.1 (0.89–1.26)	0.527
Hospital stays (days)	16.8 ± 16.0	14.3 ± 13.8	—	<0.001
Admission into ICU, *n* (%)	1786 (74.9)	2083 (70.5)	1.2 (1.10–1.41)	<0.001

AIS = abbreviated injury scale; CAD = coronary artery disease; CHF = congestive heart failure; CI = confidence interval; CVA = cerebral vascular accident; DM = diabetes mellitus; ESRD = end-stage renal disease; GCS = Glasgow Coma Scale; HTN = hypertension; ICU = intensive care unit; IQR = interquartile range; ISS = injury severity score; OR = odds ratio.

**Table 2:** Physiology and procedures performed at the emergency room in trauma patients with injury severity score equal to or more than 16.

Variables	Transfer (*n* = 2,386)	Direct (*n* = 2,955)	OR (95% CI)	*p*
Physiology at ER, *n* (%)				
GCS <13	872 (36.5)	835 (28.3)	1.5 (1.30–1.64)	<0.001
SBP <90 mm·Hg	136 (5.7)	148 (5.0)	1.1 (0.90–1.46)	0.263
HR > 100 beats/min	651 (27.3)	694 (23.5)	1.2 (1.08–1.38)	0.001
RR < 10 or >29 times/min	58 (2.4)	100 (3.4)	0.7 (0.51–0.99)	0.041

Procedures at ER, *n* (%)				
Cardiopulmonary resuscitation	10 (0.4)	40 (1.4)	0.3 (0.15–0.62)	<0.001
Intubation	95 (4.0)	545 (18.4)	0.2 (0.15–0.23)	<0.001
Chest tube insertion	119 (5.0)	193 (6.5)	0.8 (0.59–0.95)	0.017
Blood transfusion	323 (13.5)	384 (13.0)	1.0 (0.89–1.23)	0.561

ER, emergency room; CI, confidence interval; HR, heart rate; RR, respiratory rate; GCS, Glasgow Coma Scale; SBP, systolic blood pressure; OR odds ratio.

**Table 3:** Comparison of the outcome between the propensity score-matched cohorts of patients who were transferred and visited trauma centers directly.

Propensity score-matched patient cohorts					
Variables	Transfer (*n* = 2,139)	Direct (*n* = 2,139)	OR (95% CI)	*p*	Standardized difference
Male, *n* (%)	1461 (68.3)	1461 (68.3)	1.0 (0.88–1.14)	1.000	0.00%
Age (years)	53.9 ± 19.2	53.9 ± 18.6	－	0.929	−0.27%
Comorbidities					
CVA, *n* (%)	60 (2.8)	60 (2.8)	1.0 (0.70–1.44)	1.000	0.00%
HTN, *n* (%)	633 (29.6)	633 (29.6)	1.0 (0.88–1.14)	1.000	0.00%
CAD, *n* (%)	76 (3.6)	76 (3.6)	1.0 (0.72–1.38)	1.000	0.00%
CHF, *n* (%)	3 (0.1)	3 (0.1)	1.0 (0.20–4.96)	1.000	0.00%
DM, *n* (%)	311 (14.5)	311 (14.5)	1.0 (0.84–1.19)	1.000	0.00%
ESRD, *n* (%)	28 (1.3)	28 (1.3)	1.0 (0.59–1.69)	1.000	0.00%
Trauma mechanisms					
Automobile, *n* (%)	53 (2.5)	53 (2.5)	1.0 (0.68–1.47)	1.000	0.00%
Motorcycle, *n* (%)	1265 (59.1)	1265 (59.1)	1.0 (0.89–1.13	1.000	0.00%
Bicycle, *n* (%)	85 (4.0)	85 (4.0)	1.0 (0.74–1.36)	1.000	0.00%
Pedestrian, *n* (%)	70 (3.3)	70 (3.3)	1.0 (0.71–1.40)	1.000	0.00%
Fall, *n* (%)	585 (27.3)	585 (27.3)	1.0 (0.87–1.14)	1.000	0.00%
Penetrating injury, *n* (%)	5 (0.2)	5 (0.2)	1.0 (0.29–3.46)	1.000	0.00%
Strike by/against, *n* (%)	76 (3.6)	76 (3.6)	1.0 (0.72–1.38)	1.000	0.00%
ISS, median (IQR)	20 (16–25)	20 (16–25)	—	0.513	2.00%
Outcomes					
Mortality, *n* (%)	230 (10.8)	210 (9.8)	1.1 (0.91–1.35)	0.314	—
Hospital stays (days)	16.6 ± 15.8	14.7 ± 13.7	－ <0.001	—	—
Admission into ICU (%)	1581 (73.9)	1516 (70.9)	1.2 (1.02–1.33)	0.026	—

CAD = coronary artery disease; CHF = congestive heart failure; CI = confidence interval; CVA = cerebral vascular accident; DM = diabetes mellitus; ESRD = end-stage renal disease; HTN = hypertension; ICU = intensive care unit; IQR = interquartile range; ISS = injury severity score; OR = odds ratio.

## Data Availability

The data used to support the findings of this study are available from the corresponding author upon request.
